# Riparin-B as a Potential Inhibitor of AdeABC Efflux System from *Acinetobacter baumannii*

**DOI:** 10.1155/2023/1780838

**Published:** 2023-04-08

**Authors:** Patrícia Virna Sales Leão, Ana Laura da Silva Ferreira, Felipe Araújo de Alcântara Oliveira, Avilnete Belém de Souza Mesquita, José de Sousa Lima-Net, Stanley Juan Chavéz Gutierrez, Carlos Emídio Sampaio Nogueira, Natália Cruz-Martins, Daniel Dias Rufino Arcanjo, Humberto Medeiros Barreto, Josie Haydée Lima Ferreira

**Affiliations:** ^1^Laboratory of Research in Microbiology, Department of Parasitology and Microbiology, Federal University of Piaui, Teresina, Piauí, Brazil; ^2^Department of Pharmacy, Federal University of Piauí, Teresina, Piauí, Brazil; ^3^Department of Biological Chemistry, Regional-University of Cariri, Crato, Ceará, Brazil; ^4^Faculty of Medicine, University of Porto, Alameda Prof. Hernâni Monteiro, Porto 4200-319, Portugal; ^5^Institute for Research and Innovation in Health (i3S), University of Porto, Porto 4200-135, Portugal; ^6^Laboratory of Functional and Molecular Studies on Physiopharmacology (LAFMOL), Department of Biophysics and Physiology, Federal University of Piaui, Teresina, Piauí, Brazil

## Abstract

*Acinetobacter baumannii* is an important opportunistic pathogen that causes serious health-related infections, especially in intensive care units. The present study aimed to investigate the antimicrobial activity of Riparin-B (Rip-B) alone and in association with norfloxacin against multidrug-resistant clinical isolates of *A. baumannii*. For this, the minimum inhibitory concentrations were determined by the microdilution method. For the evaluation of resistance-modulating activity, MIC values for antibiotics were determined in the presence or absence of subinhibitory concentrations of Rip-B or chlorpromazine (CPZ). The AdeABC-AdeRS efflux system genes from these isolates were detected by PCR. Docking studies were also carried out to evaluate the interaction of Riparin-B and the AdeABC-AdeRS efflux system. The study was conducted from 2017 to 2019. The results showed that Rip-B showed weak intrinsic activity against the strains tested. On the other hand, Rip-B was able to modulate norfloxacin's response against *A. baumannii* strains that express efflux pump-mediated resistance. Docking studies provided projections of the interaction between Rip-B and EtBr with the AdeB protein, suggesting that Rip-B acts by competitive inhibition with the drug. Results found by in vitro and in silico assays suggest that Rip‐B, in combination with norfloxacin, has the potential to treat infections caused by multidrug-resistant *A. baumanni* with efflux pump resistance.

## 1. Introduction

Infections caused by multidrug-resistant micro-organisms are a current problem of public health all over the world and they have increased the morbidity and mortality rates in the population [1, 2]. Previous data from the National Network for Monitoring Microbial Resistance in Health Services, Brazil, showed that *Acinetobacter* spp. is the most critical of all the types, including multidrug-resistant bacteria, which are particularly dangerous in hospital areas, retirement houses, and among patients whose care demands the use of ventilators and intravenous catheters [3].

The *A. baumannii* is an aerobic, nonfermented, Gram-negative, coccobacillus labeled as an opportunistic pathogen widely associated with infection outbreaks related to health assistance, verified in intensive center unity environments [4]. Infections caused by that pathogen are intricately linked to pneumonia, septicemia, meningitis, urinary tract infections, surgical wounds, previous antibiotic therapy, burns, and immunosuppression diagnoses [5].

*A. baumannii* shows unconventional resistance to multiple drugs, and it may also bear countless protection mechanisms against most regular antibiotic substances used in its treatment [6]. This resistance might come from uncounted mechanisms, intrinsic or acquired because of an overproduction of efflux pumps, permeability reduction of the outer membrane, amendment of the target site, and production of beta-lactamases [7]. Similar mechanisms are also verified for resistance to biocides acquired by clinical isolates of *A. baumannii* [8].

The search for alternative therapies to resistant micro-organisms inspires research on the microbicidal potential of some plants and its metabolites [9, 10] such as the substance alcamida, separated from the unripe fruit of *Aniba riparia* (Nees) Mez belonging to *Lauraceae* family. Riparins I, II, and III are substances that occur naturally isolated from *A. riparia*. These chemical compounds derived from Riparins showed diverse biological activities. In addition to the natural occurrence of molecules originating in *A. riparia*, synthetic Riparins such as Riparin-B (Rip-B) was obtained by the Schotten–Bauman reaction [11].

Previous research carried out by our group pointed out that Rip-B was enhanced the action of norfloxacin and ciprofloxacin by inhibition of NorA efflux pump of *Staphylococcus aureus* [12]. This result motivated us to investigate if Rip-B could modulate the resistance of clinical isolates of *A. baumanni* carrying the AdeABC-AdeRS efflux system.

## 2. Results

### 2.1. Intrinsic Antimicrobial Activity of Riparin-B

In the present study, the synthetic derivative Rip-B (Figure 1) was investigated for its potential antimicrobial activity against different *A. baumannii* strains isolated from an urgency hospital of Teresina, Piauí, Brazil. Rip-B is a nonheterocyclic alkaloid, more specifically, a natural alkamide. It is formed from the union of tyramine, a phenylalanine and benzoic acid. It adds a substitution in the ring of benzoic acid, adding a hydroxyl, and the tyramine ring presents a methyl linked to oxygen forming an ether function.

Our results showed that Rip-B did not have intrinsic antimicrobial activity against multidrug-resistant *A. baumannii* strains tested (Table 1).

### 2.2. Evaluation of the Drug-Resistance Modulation

In the tests where Rip-B was added at subinhibitory concentration there was a significant reduction in the MIC values for norfloxacin, as it happens when a known efflux pump inhibitor (CPZ) is put in combination with norfloxacin (Figure 2). These results indicate that Rip-B is a modulating agent of the drug resistance in *A. baumannii* strains.

Ethidium bromide (EtBr) is a genotoxic dye that intercalates into DNA double-helix leading, to DNA damage and cell death, and the only known mechanism of resistance to EtBr in bacteria is mediated by the efflux pump [13]. Thus, this intercalating agent has been used as an indicator of the resistance mediated by efflux pumps [14]. In the present study, the modulating effect of Rip-B on the resistance to EtBr was verified only in the strains expressing resistance mediated by efflux pump phenotype (Figure 3). These results are strong evidence that modulating of the antibiotic resistance by Rip-B could be due to efflux pump inhibition.

### 2.3. Antimicrobial Susceptibility Profile and Distribution of the AdeABC-AdeRS Efflux System Genes

Table 2 shows the presence of genes from the AdeABC-AdeRS efflux system among the resistant strains of *A. baumannii* multidrug (MDR) used in this study. It was observed that the strains tested have genes from the AdeABC-AdeRS efflux system. The three strains also amplified the *oxa*-*51* gene, confirming that it is *A. baumannii*. Table 2 also provides information on the resistance profile of the clinical isolates of *A. baumanii*. All *A. baumannii* clinical isolates tested were multidrug-resistant (MDR) and were resistant to norfloxacin.

### 2.4. Docking

To the best of our knowledge, there are no docking studies involving Rip-B on the AdeABC efflux pump. Thus, to check if this substance could indeed act as an AdeABC inhibitor and to get some insights on the inhibition mechanism, we have carried out the docking of Riparin-B and the known substrate EtBr with the AdeABC structure as a target. The AdeABC efflux system is comprised of three parts: the AdeA periplasmic protein, the AdeB efflux pump protein, and the AdeC outer membrane protein. AdeB has a 3-fold symmetrical structure with two periplasmic multidrug binding sites: distal and proximal. A drug supposedly enters the protein through a periplasmic cleft and binds to the proximal site, passes through a gate loop (G-loop), and is then delivered to the distal site for extrusion [15]. These sites are shown in Figure 4, labeled *P* (proximal) and *D* (distal). Figure 4 displays the best poses of both EtBr and Rip-B docked on the binding site of the AdeABC efflux pump. A 2D protein-ligand diagram for EtBr is provided in Figure 5 and 2D protein-ligand diagram for Riparin-B is provided in Figure 6.

## 3. Discussion

Due to the high prevalence of infections caused by multidrug-resistant *A. baumannii*, mainly in hospital environments, the research of new antimicrobial agents effective against this pathogen has been considered as a priority. To contribute to this context, we analyzed the intrinsic antimicrobial activity of Rip-B against *A. baumannii* clinical isolates, as well as its modulating activity on the resistance to norfloxacin. The molecular and susceptibility profile characterization of the clinical samples used in this study shows a multidrug-resistance profile and confirms the presence of genes from the AdeABC efflux system. Our previous study reported a high percentage of extremely drug-resistant (XDR) strains (81.1%) that was verified among *A. baumannii* clinical isolates at a northeast Brazilian Emergency Hospital, with greater prevalence of resistance to gentamicin (98.0%), ceftriaxone (94.3%), ceftazidime (92.0%), ciprofloxacin (90.5%), and levofloxacin (90.5%) [16]. Several studies report the prevalence of multi-resistant and extremely resistant clinical isolates among strains of hospital origin, showing a great diversity of mobile genetic elements and the ability to acquire and expand expressed of the antimicrobial resistance factors [17–21].

Rip-B did not show intrinsic antimicrobial activity; however, enhanced the activity of norfloxacin against clinic strains of *A. baumannii*, showing that it could be useful as an adjuvant of norfloxacin in the treatment of infections caused by multidrug-resistant *A. baumannii*. The antibacterial activity of natural Riparins I, III, and XII isolated from *A. riparia* against multidrug-resistant *S. aureus* and *E. coli* strains has already previously reported [22]. Moreover, while the synthetic analog Rip-E showed a good antibacterial activity against *S. aureus* strains, the synthetic derivative Rip-B was inactive against *S. aureus* [11]. In the present study, we also verified that Rip-B was inactive against all *A. baumannii* strains tested once MIC values were found higher than 1000 *μ*g/mL (Table 1) which is considered as clinically insignificant [23]. These results show that Rip-B it is not recommended for use as an antimicrobial agent.

The natural Rip-III isolated from *A. riparia* was able to induce plasmid elimination in *S. aureus* strains changing the Penicillin resistance phenotype to sensitive [24]. Furthermore, Rip-B was reported as being an inhibitor of the NorA, an efflux pump of *S. aureus* belonging to the Major Facilitator Family [12]. These studies motivated us to investigate if Rip-B were able to potentiate the norfloxacin activity against *A. baumannii* strains expressing-resistance mediated by efflux pump phenotype, with the goal of suggesting a possible use of Rip-B as an adjuvant of this antibiotic in the treatment of *A. baumannii* infections. The results in Figure 2 suggest that Rip-B inhibits the efflux pump mechanism by decreasing MIC values for norfloxacin, modulating the action of this drug in the clinical strains of *A. baumannii*. This hypothesis was corroborated by results obtained for the known NorA inhibitor CPZ [25] that also modulated the antibiotic resistance in the *A. baumanii* strains expressing the AdeABC-AdeRS genes.

Since the presence of efflux pumps is the only known resistance mechanism for EtBr, assays using ethidium bromide (Figure 3) reinforce the evidence that the modulation of norfloxacin resistance by Rip-B occurs due to efflux inhibition. In fact, a previous study reported that Rip-B is an inhibitor of NorA, a proton-motive force dependent efflux pump of *S. aureus* belongs to the major facilitator superfamily (MFS), able to compete with antibiotic by the same binding pocket formed by ILE19, ILE23, PHE26, PHE47, ALA48, GLN51, MET109, THR113, SER133, ILE136, THR211, ARG310, ILE313, THR314, ASN332, SER333, THR336, SER337, ASN340, and PHE341 [12]. NorA extrudes hydrophilic fluoroquinolones, such as norfloxacin and Ciprofloxacin, and other biocides as quaternary ammonium compounds and EtBr [26].

In *A. baumannii*, resistance to Norfloxacin can be mediated by the multidrug efflux pump AdeABC, a proton-motive force dependent efflux pump belongs to the Resistance and Nodulation Cell Division (RND) [27–31]. It is observed that in the strain HUT90 the presence of all genes of the AdeABC-AdeRS complex was detected, while in strains HUT 89 and 105 the presence of the AdeB gene was detected, however, there was no amplification of the regulatory AdeR and AdeS genes (Table 2). High frequencies of overexpression of AdeABC genes were reported for clinical isolates of *A. baumannii* from Brazil [31] and France [32]. However, the distribution of genes in this system was not homogeneous among strains. Frequencies of 92.4%, 98.5%, 92.4%, 90.9%, and 92.4%, respectively, for the AdeA, AdeB, AdeC, AdeR, and AdeS genes were found in *A. baumannii* strains resistant to carbapenems, meanwhile in strains sensitive to carbapenems, such as 105 strain tested in the present study, the presence of AdeRS genes occurred in 50–55% of the strains evaluated [33]. A previous study also point out that the expression of the AdeA, AdeB, and AdeC genes are inconsistent and that despite variations in detection rates, there is a predominance of amplification of the AdeB gene in clinical isolates of *A. baumannii* [28].

Another important point to consider is that functional mutations have been found in conserved domains of AdeRS in all strains that overexpress AdeABC [28, 34]. Furthermore, it is known that functional mutations in the insertion sequence (IS) in AdeRS can also affect the regulation of the AdeABC system, leading to overexpression of the system [35]. The way in which the AdeR and AdeS genes regulate the overexpression of the AdeABC system is not fully understood. The analysis of the interaction between AdeR and AdeABC by electrophoresis mobility shift rehearsal and found that the promoters AdeR and AdeABC did not interact [36]. Even if AdeS was present, AdeR was not found to link to the promoting region of AdeABC. In this way, it is known that AdeRS that regulates the expression of AdeABC is defined, but the mode of action is still difficult to specify. In addition, the regulation of AdeABC gene expression is complex. Under some conditions, the insertion of ISAbaI does not lead to overexpression of this pump [37], indicating that other regulators may be involved. Lin et al. [38] also showed that the other two-component system, BaeSR, can regulate AdeA and AdeB. Thus, in strains 89 and 105, regulation of the overexpression of the AdeABC genes may be occurring by mutation in the amplification regions or by another mechanism not yet known. Multidrug-resistant strains overexpressing efflux pumps are able to extrude this antibiotic reducing its intracellular concentrations. Thus, it is possible that the strains tested in the present study, even with different genetic profiles, could overexpress AdeABC that were inhibited by Rip-B. In its turn, inhibition of efflux pumps by Rip-B could lead to a higher antibiotic accumulation in periplasm or cytoplasm where antibiotic targets are located enhancing their activity.

Previous study documented that both *Holarrhena antidysenterica* extract and conessine, a steroidal alkaloid compound, could restore antibiotic activity due to interference with the AdeIJK pump in *A. baumannii*, not interfering with the AdeABC pump [39]. However, the presence of AdeABC efflux pump genes in the strains of clinical origin in the study had not been confirmed, unlike what was done in this study. The same alkaloid, conessine, was shown to be effective as an efflux pump inhibitor in *Pseudomonas aeruginosa* [40]. Both studies indicated the potential of an alkaloid product as an inhibitor of the homologous resistance-nodulation-splitting (RND) family.

Docking studies of Rip-B on the NorA efflux pump of *Staphylococcus aureus* were already reported by Costa et al. [12]. Figure 4 shows the possible binding sites of a drug with the AdeB protein, highlighting the proximal and distal sites. As reported by Su et al. [15], residues Phe179, Phe277, Ile607, and Trp610 create a hydrophobic patch that could be connected to the stabilization of substrates. The best pose of EtBr (with a binding energy of −7.3 kcal/mol) makes close contact with Trp610 and to some residues of the G-loop, such as Gly611, Phe612, and Gly614. It also interacts through a hydrogen bond (2.24 Å) with Asp83. Rip-B also bind to this region (with binding energy of −7.3 kcal/mol), in-between both binding sites, interacting with residues 610 through 615 of the G-loop. There is also a hydrogen bond with Gly615, and close contacts with several residues, with two in particular: Thr91 and Ser134. It is reported that the antibiotic gentamicin interacts with these residues and ciprofloxacin binding site overlaps with that of gentamicin (10.1128/mBio.01295-19). Interestingly, Tyr77, Thr91, and Ser134 are conserved residues between AdeB and the MexY pump. There's reason to believe, therefore, that these residues play a significant role in drug recognition. As both EtBr and Rip-B bind to the same region of the binding site one could argue that Rip-B could act as a competitive inhibitor, preventing the extrusion of drugs as norfloxacin and EtBr. Binding near the G-loop, Rip-B could, for instance, hinder the passing of drugs from the proximal to the distal site. Its preferred site also overlaps with that of antibiotics such as gentamicin. Thus, they could also be expelled in place of the antibiotic, acting as a competitive inhibitor.

## 4. Materials and Methods

### 4.1. Strains and Chemicals

Evaluation of the Rip-B antimicrobial activity was performed against multidrug-resistant *A. baumannii* strains isolated from patients attended in an urgency hospital from Teresina, Piauí, Brazil. The isolates were collected from cultures of respiratory tract specimens (HUT 89 *e* HUT 90) and spinal cerebral fluid aspirate (HUT 105). Bacterial strain isolation was performed in blood agar followed by subculture in MacConkey Agar (Sigma–Aldrich) using duplicates. Bacterial strain identification was performed using the BD PHOENIX 5.1 automation method (Becton Dickison Sparks, MD 21152, USA) and confirmed on blaOXA-51 polymerase chain reaction (PCR), as described in item 4.6.

Assays for evaluation of the modulating effect of Rip-B on the antibiotic resistance were performed with multidrug-resistant *A. baumannii* (according to item 4.2) previously screened to resistance mediated by efflux pump phenotype with carbonylcyanide m-chlorophenylhydrazone (CCCP, Sigma–Aldrich), as described in item 4.3. For a comparison, also were conducted assays with strains expressing resistance not mediated by efflux pumps. Bacterial strains were maintained on Brain Heart Infusion Agar (BHIA, Himedia, India) slants at 4°C, and prior to the assay the cells were grown overnight at 37°C in Brain Heart Infusion (BHI, Himedia, India). Norfloxacin (Nor), ethidium bromide (EtBr), and chlorpromazine (CPZ) were obtained from Sigma Chemical Corp., St. Louis. Nor was dissolved in a mixture of 1 M NaOH and sterile distilled water (1 : 9 proportion). EtBr and CPZ were dissolved in sterile water. N-[2-(3,4-dimethoxyphenyl)ethyl]-benzamide (Riparin-B, Brazil) was prepared in dimethyl sulfoxide (DMSO, Merck) and then diluted with sterile water.

### 4.2. Antimicrobial Susceptibility Testing

Antimicrobial susceptibilities for isolates were determined initially using the BD PHOENIX 5.1 automation method (Becton Dickison Sparks, MD 21152, USA). The resistance profile of the isolated strains was confirmed by the diffusion method according to the Clinical and Laboratory Standards Institute - CLSI [41]. The tested antimicrobials were gentamycin (GEN), ceftriaxone (CRO), ciprofloxacin (CIP), ceftazidime (CAZ), levofloxacin (LEV), amikacin (AMI), cefepime (CPM), piperacillin-tazobactam (PPT), meropenem (MER), imipenem (IPM), sulfamethoxazole-trimethoprim (SUT), tigecycline (TIG), and colistin (COL) (Laborclin, Brazil). *Pseudomonas aeruginosa* ATCC 27853 and *A. baumanii* NCTC 13304 (Controlab, Brazil) were used as controls.

### 4.3. Determination of the Occurrence of Resistance Mediated by Efflux Pump Phenotype

To verify the occurrence of efflux pump-mediated resistance, MIC values of amikacin, ceftazidime or norfloxacin were determined in the presence or absence of a carbonyl cyanide m-chlorophenylhydrazone (CCCP, Sigma–Aldrich) solution at the subinhibitory concentration. CCCP is a decoupler from oxidative phosphorylation that interrupts the proton gradient of membranes. Microtitration plates were incubated at 37°C for 24 hours, and following this time 20 *μ*l of a 0.01% (w/v) aqueous Resazurin sodium (Sigma–Aldrich) solution was added to each well. These plates were incubated for 1 hour at room temperature, where following this period a reading was performed taking into account that a change in coloration from blue to pink indicated the occurrence of bacterial growth due to resazurin reduction [42, 43]. As a criterion for classifying the occurrence of resistance mediated by the efflux pump phenotype, a minimum of a 2-fold antibiotic MIC reduction in the presence of CCCP was necessary [22].

### 4.4. Assays for Evaluation of the Intrinsic Antimicrobial Activity

Stock solutions of Rip-B or CPZ were prepared in DMSO (Merck), followed by dilution in sterile distilled water to a final concentration of 1024 *μ*g·mL^−1^. Minimal inhibitory concentrations (MICs) were determined by microdilution assay in BHI broth with bacterial suspensions of approximately 105 CFU·mL^−1^ and concentrations of Rip-B (or CPZ) solution ranging from 8 to 512 *μ*g·mL^−1^. Microtiter plates were incubated at 37°C for 24 h, and then 20 *μ*L of resazurin (0.01% w/v in sterile distilled water) was added to each well to detect bacterial growth by a visual color change from blue to pink as described above.

### 4.5. Assays for Evaluation of the Drug-Resistance Modulation

To evaluate if Rip-B was able to modulate antibiotic resistance in *A. baumannii* strains expressing or not resistance mediated by efflux pump phenotype, MIC value for norfloxacin was determined in the presence or absence of Rip-B solution at subinhibitory concentration (MIC 1/8). Antibiotic concentrations ranged from 0.125 to 128 *μ*g·mL^−1^. Microtiter plates were incubated at 37°C for 24 h and readings were performed with resazurin as described above. To verify if the drug-resistance modulation occurred due to efflux pump inhibition, modulation assays were performed replacing antibiotics by EtBr, which is a known substrate of efflux pumps [13]. Control assays were also performed replacing Rip-B y CPZ (Sigma–Aldrich) which is a known efflux pump inhibitor [19]. Microtiter plates were incubated at 37°C for 24 h, and then 20 *μ*L of resazurin (0.01% w/v in sterile distilled water) was added to each well to detect bacterial growth by a visual color change from blue to pink as described above.

### 4.6. Identification of the AdeABC-AdeRS Efflux System Genes

Bacterial DNA was extracted from *A. baumannii* isolates by boiling. PCR was performed using Taq DNA Polymerase (Ludwig Biotec). The primes used were: OXA-51F: TCCAAATCACAGCGCTTCAAAA; OXA-51R: TGAGGCTGAACAACCCATCCA; AdeA F: GAGGTGGCAAGACTCAAAGTTC; AdeA F: GAGGTGGCAAGACTCAAAGTTC; AdeA R: GCTAGAGCCTGACGATACTGAGC; AdeB F: TACCGGTATTACCTTTGCCGGA; AdeB R: GTCTTTAAGTGTCGTAAAAGCCA; AdeC F: ACAATCGTATCTCGTGGACTC; AdeC R: TAGAAACTGGGTTATTGGGGT; AdeR F: ACTACGATATTGGCGACATT; AdeR R: GCGTCAGATTAAGCAAGATT; AdeS F: TTGGTTAGCCACTGTTATCT; AdeS R: AGTGGACGTTAGGTCAAGTT [44–46]. PCR was performed in a 25 *μ*L reaction mixture containing 1 *μ*L primer, 1 *μ*L Taq polymerase (Ludwig Biotec), 3 *μ*L DNA template, 3.0 mM MgCl2, 2.5 *μ*L 10 × buffer, 0.2 mM dNTPs, and nuclease-free water. Amplification conditions consisted of denaturation at 94°C for 5 min and 30 cycles of denaturation at 94°C for 1 min, annealing at 56°C for 30 s and extension at 72°C for 1 min, with a final extension at 72°C for 10 min. PCR products were detected in 2% agarose gel.

### 4.7. Docking Procedure

The structure for the AdeABC efflux pump was downloaded from the RCSB.org [47] site (PDB-ID: 6OWS). The structure was uploaded to the MolProbity Server for protonation [48]. Ligands were optimized using the Gaussian 09 Program [49]. Initial structures were created in the GaussView module and were then optimized using the PM6 forcefield. Partial Gasteiger charges were added to the protein (although Autodock Vina ignores it) and to the ligand atoms using the AutoDock Tools interface [50], nonpolar hydrogen atoms were mixed while all other parameters were kept at their default values. Docking procedure was carried out using the Autodock Vina software [51]. The docking poses were chosen based on the best binding score.

### 4.8. Statistical Analysis

Experiments were performed in triplicate and results were normalized by calculation of geometric mean values. The error deviation and standard deviation of the geometric mean were revealed. Statistical analyzes were performed using GraphPad Prism, version 5.02. Differences between treatment with antibiotics (or EtBr) alone or associated with Rip-B or CPZ were examined using one-way analysis of variance (ANOVA). The differences mentioned above were analyzed by Bonferroni posttest and *p* < 0.05 were considered statistically significant.

## 5. Conclusions

The combination of antibiotics with efflux pump inhibitors may be a promising strategy for the treatment of infections caused by multidrug-resistant A. baumannii. Results obtained in the present study showed that Rip-B was inactive against *A. baumannii* strains. However, Rip-B was able to increase the activity of norfloxacin against strains of *A. baumannii* that exhibit efflux pump-mediated resistance. The results obtained through Rip-B/EtBr association tests suggested that the increase in antibiotic activity probably involves the inhibition of overexpressed efflux pumps in the strains tested. The clinical isolates of *A. baumannii* MDR had genes for the AdeABC-AdeRS efflux system, with the AdeB gene present in all tested isolates. Docking studies show the interaction of Rip-B and EtBr with the proximal and distal sites of the AdeB protein, suggesting that Rip-B could act as a competitive inhibitor for both norfloxacin and EtBr, preventing the passage of these compounds from the proximal to the distal site. As a limitation, the present study did not investigate if Rip-B could inhibit the expression of the AdeABC-AdeRS genes. Thus, Rip-B could be applied as an adjuvant of norfloxacin in the treatment of infections caused by multi-resistant strains of *A. baumannii* with resistance by efflux pumps. However, *in vivo* preclinical studies will be needed to verify if Rip-B could enhance the norfloxacin activity against *A. baumannii* strains expressing AdeABC-AdeRS genes genes in animal models experimentally infected.

## Figures and Tables

**Figure 1:** Chemical structure of the Riparin-B (N-[2-(3,4-dimethoxyphenyl)ethyl]-benzamide).

**Figure 2:** MIC values for norfloxacin (Nor) found in the absence or presence of the Rip-B or chlorpromazine (CPZ) against clinical isolates of *A. baumannii* expressing resistance mediated by efflux pump phenotype. Each result is the geometric mean of three simultaneous experiments. (^*∗∗∗∗*^) Statistically significant values (*p* < 0.0001).

**Figure 3:** MIC values for ethidium bromide (EtBr) found in the absence or presence of the Rip-B or chlorpromazine (CPZ) against clinical isolates of *A. baumannii* expressing resistance mediated by efflux pump phenotype. Each result is the geometric mean of three simultaneous experiments. (^*∗∗∗∗*^) Statistically significant values (*p* < 0.0001).

**Figure 4:** (Left) the binding sites of the AdeABC efflux pump. The distal and proximal sites are labeled as *D* and *P*, respectively. (Right) the best poses of EtBr (yellow) and Rip-B (pink).

**Figure 5:** 2D protein-ligand diagram for ethidium bromide (EtBr).

**Figure 6:** 2D protein-ligand diagram for ethidium bromide (EtBr).

**Table 1:** Geometrical means of the minimum inhibitory concentration (MIC) of Riparin-B (Rip-B) against clinical isolates of *Acinetobacter baumannii* resistant to norfloxacin.

Strains	MIC (*μ*g/mL)	Inhibitory effect
HUT-89	1024	No activity
HUT-90	1024	No activity
HUT-105	1024	No activity

**Table 2:** Distribution of Ade efflux pump genes in the MDR *A. baumannii* isolates in this study.

Isolates	OXA-51	AdeA	AdeB	AdeC	AdeR	AdeS	Antimicrobial resistance
HUT89	+	+	+	+	−	−	CAZ, CPM, CRO, CIP, NOR, LEV, IPM, MER, GEN, AMI, PPT, and SUT *e* TIG.
HUT90	+	+	+	+	+	+	CAZ, CPM, CIP, NOR, LEV, IPM, MER, GEN, AMI, and PPT *e* TIG.
HUT105	+	−	+	+	−	−	CAZ, CPM, CRO, CIP, NOR, LEV, GEN, AMI, PPT, and SUT *e* TIG.

Ceftazidime (CAZ), cefepime (CPM), ceftriaxone (CRO), ciprofloxacin (CIP), norfloxacin (NOR), levofloxacin (LEV), imipenem (IPM), meropenem (MER), gentamycin (GEN), amikacin (AMI), piperacillin-tazobactam (PPT), cefepime (CPM), sulfamethoxazole-trimethoprim (SUT), tigecycline (TIG).

## Data Availability

The data supporting the current study are given in the article.

## Additional Points

Sample of the Riparin-B and clinical strains of the *A. baumanii* are available from the authors.
